# Health Impact Assessment of Short-Term Exposure to Particulate Matter (PM_10_) in Northern Thailand

**DOI:** 10.1155/2023/1237768

**Published:** 2023-05-29

**Authors:** Pakaporn Ngamsang, Teerachai Amnuaylojaroen, Nichapa Parasin, Sittichai Pimonsree

**Affiliations:** ^1^School of Energy and Environment, University of Phayao, Phayao 56000, Thailand; ^2^Atmospheric Pollution and Climate Change Research Units, School of Energy and Environment, University of Phayao, Phayao, Thailand; ^3^School of Allied Health Science, University of Phayao, Phayao 56000, Thailand

## Abstract

In northern Thailand, in recent decades, particulate pollution from the burning of biomass has become a serious issue with toxicological implications for human health, especially during the winter months of January to April. The purpose of this study was to explore short-term exposure to particulate matter (PM_10_) in northern Thailand. The high PM_10_ concentration in 2012 was used as a case study. We used the EPA's Benefits Mapping and Analysis Program-Community Edition (BenMAP-CE) for the health impact assessment, along with ground-based measurement data. The annual average observed PM_10_ concentration was in the range of 43–61 *μ*g/m^3^, with a maximum observed PM_10_ concentration of 300 *μ*g/m^3^ in March. We then assessed the impacts of PM_10_ exposure in northern Thailand. When the PM_10_ concentration was reduced to 120 *μ*g/m^3^, the undesirable effects on respiratory mortality decreased by 5%–11%. When the concentration of PM_10_ was reduced to 45 *μ*g/m^3^, the deleterious effects on respiratory mortality decreased by 11–30%. In conclusion, adherence to the WHO-AQG, particularly for PM_10_ (45 *μ*g/m^3^), tends to result in considerable reductions in respiratory disease mortality in northern Thailand.

## 1. Introduction

Air pollution is a major problem and has severe toxicological effects on human health and the ecosystem [1, 2]. It is widely recognized that air pollution contributes to the onset of illnesses such as infectious diseases, inflammatory disorders, and cancer [3–6]. It is also responsible for millions of deaths worldwide each year [7–10].

In recent decades, biomass burning has been a major source of air pollution in northern Thailand, particularly between January and April [11–13]. In addition, significant haze episodes in this region have become increasingly severe and frequent in recent years due to increased particle pollution. Factors contributing to northern Thailand's air quality problems include emissions from extensive biomass burning and human activities from both domestic and neighboring countries, which release particle pollution [11, 14–16]. Moreover, the combination of topographic and meteorological characteristics stimulates environmental conditions that are conducive to and which contribute to the air pollution problem in northern Thailand. People in northern Thailand are subjected to annual periods of biomass burning from agricultural waste and forestry inside and outside Thailand (in neighboring countries), resulting in unusually high particulate pollution from January to April each year [17–21].

Several unfavorable health consequences can arise from exposure to high amount of air pollution. A considerable number of studies of short-term exposure to air pollution have examined the associations between low air quality levels and daily variability in death rates [22, 23]. High levels of particulate matter (PM) potentially pose a threat to human health because, based on their size, the inhaled particles may reach critical depths in the lungs, causing detrimental health effects. Several studies have revealed a correlation between high levels of particulate matter and an increase in respiratory and cardiovascular pathologies; for example, the studies conducted by [17, 24–27] and Kelly et al. [28] suggested that PM_10_ levels below the EU Directive 2008/50/EC daily limit (50 *μ*g/m^3^) are related to an elevated risk of acute cardiovascular events. In addition, the International Agency for Research on Cancer listed outdoor air pollution and particle matter as carcinogenic. Although PM_10_ air pollution impacts the entire population, it has been established that children, elderly adults, and those with preexisting health conditions are more susceptible to acquiring specific illnesses [29, 30]. Moreover, PM_10_ has significant short-term health impacts. Years of life lost (YLL) due to nonaccidental fatalities increased by 1.23 (95% CI: 0.15, 2.31), 2.18 (0.35, 4.01), 0.28 (1.27, 1.82), 1.06 (1.25, 3.37), and 2.00 (0.20, 3.79) for every 10 *μ*g/m^3^ increase in PM_10_ at lag 0-1 day for the full year, winter, spring, summer, and autumn, respectively [31]. During a study period (2006–2010) in major Chinese cities, a 10 *μ*g/m^3^ increase in monthly PM_10_ concentration was linked to a 1.05% increase in the adult respiratory death rate [32]. In Shenzhen, China, the excess risk of all-cause death with an increase in PM_10_ of 10 g/m^3^ was 0.61% (95% confidence interval (CI): 0.50–0.72) [33]. These studies suggest that short-term PM_10_ exposure has significant public health impacts.

A health impact assessment (HIA) is a robust approach for evaluating the adverse health effects of air pollution on a population, particularly on socioeconomically deprived people [34]. Utilizing quantitative, qualitative, and participatory approaches, this strategy is applicable to numerous economic sectors. The Benefits Mapping and Analysis Program-Community Edition (BenMAP-CE) of the Environmental Protection Agency is a helpful tool for HIA. It is typically used to assess the impact of air pollution on human health. For example, Mueller et al. [35] used the PM_2.5_ concentrations observed from ground-based measurements in Thailand from 1996 to 2016 to estimate the economic and health impacts of long-term exposure to ambient PM_2.5_ in the Thai population using BenMAP. Fold et al. [36] used BenMAP to examine annual morbidity associated with PM_2.5_ in Bangkok, Thailand, from 2012 to 2018. Nguyen et al. [37] used BenMAP to estimate the public health and economic impacts of PM_2.5_ exposure in Mainland Southeast Asia (MSEA).

To elucidate and emphasize the disease burden caused by particle air pollution, we reveal the findings of a health impact assessment (HIA) conducted using BenMAP-CE in eight northern Thai provinces. The HIA generated estimates of the amount of respiratory illness mortality in northern Thailand attributable to PM_10_ exposure. First, we analyzed a situation in which the PM_10_ daily mean was reduced by 120 *μ*g/m^3^, and then, we described a scenario in which the PM_10_ daily mean was reduced to the WHO-AQ standard (45 *μ*g/m^3^).

## 2. Methodology

To study the effects of PM_10_ on the health of people in northern Thailand, we used daily PM_10_ concentration data from eight ground-based measurement sites from the Thai Pollution Control Department in the year 2012 as input data for the U.S. Environmental Protection Agency's Benefits Mapping and Analysis Program-Community Edition (BenMAP-CE). Two hypothetical scenarios for reducing PM_10_ concentration were evaluated in this study. In both scenarios, the excess O_3_ concentration was rolled back to the EPA's standard level of ≤0.070 ppm (using the percentage rollback method in BenMAP-CE). In the first scenario, the excess PM_10_ concentration was rolled back to the daily Thailand air quality guidelines (120 *μ*g/m^3^); meanwhile, in the second scenario, it was rolled back to the daily WHO air quality guidelines (45 *μ*g/m^3^).

### 2.1. General Information of BenMAP-CE

BenMAP is an effective HIA tool. It was published in 2003 and is the primary tool used by the United States Environmental Protection Agency (EPA) to quantify the health and economic benefits of achieving the future National Ambient Air Quality Standards (NAAQS) [38, 40]. BenMAP-CE is identical to the previous version utilized by the United States Environmental Protection Agency for a range of strategy assessments.

### 2.2. Study Area and Air Pollution Data

In this study, we used the observed PM_10_ data from eight locations (Lampang, Chiang Mai, Nan, Lamphun, Phrae, Chiang Rai, Phayao, and Mae Hong Son) from the Thai Pollution Control Department in northern Thailand between the years 2010 and 2020 (Figure 1). The quality of the data was analyzed using the standard method, as described by Wong et al., [41]. The percentage of missing data was in the range of 0.80%–20.10% during the years 2010–2020 (Table 1). We found a number of days on which the Thailand 24-hour guideline (120 *μ*g/m^3^) was exceeded, particularly in the years 2010, 2011, and 2012, as well as in 2016, 2019, and 2020. The daily average of PM_10_ concentration in northern Thailand was in the range of 36.1–47.5 *μ*g/m^3^ during the years 2010 and 2020. The highest number of days exceeding Thailand's air quality standard and mortality rate were 175 days and 0.32, respectively, in 2012, with an acceptable missing data rate of 8.50% and an average PM_10_ of 47.5 ± 4.4 *μ*g/m^3^ in northern Thailand. As a result, we selected the year 2012 as the case study in this work.

### 2.3. Estimating Human Health Impacts

To estimate the impacts of PM_10_ on human health, equation (1) was used to calculate the number of individuals who avoided death (US EPA 2018):

(1) $$\begin{array}{c} ∆Y=Yo\left(1-e^{-\beta ∆PM}\right)*Pop\text{,} \end{array}$$

where ΔPM is the change in air quality, i.e., the difference between the baseline air pollution level and the air pollution level after some controls. Pop is the number of people in northern Thailand who are at risk of becoming exposed to PM_10_ and who are aged 18 and above, as listed in Table 2. Meanwhile, the health effect estimate (*β*) is based on the following equation:

(2) $$\begin{array}{c} \beta =\log\left(\frac{epide\;miology}{∆PM}\right)\text{,} \end{array}$$

where *β* is a percentage change in the risk of significant health effects produced by a one-unit increase in ambient air pollution.

In terms of epidemiological studies linking short-term PM_10_ exposure to mortality in northern Thailand, the epidemiology was derived from the relative risk (RR) value taken from a previous study by [42], as given in Table 2. They performed a cross-sectional study between March 2016 and March 2018 (a total 761 days) in Chiang Mai province in northern Thailand. A time-series analysis was used to examine associations between air pollution levels and changes in mortality (specifically, nonaccidental mortality and cardiopulmonary diseases) for a study population. To assess the lag structure between daily average concentrations of PM_10_ and daily respiratory disease, they examined separate models for each lag from 0 to 7 days prior to the events. A lag time of zero (lag 0) was defined as same-day exposure to PM_10_. Finally, the adjusted RRs with 95% confidence intervals (CI) from regression analysis were estimated for each 10 *μ*g/m^3^ increment of PM_10_ [43]. In this study, we used the RR values at lag 6, which is the statistical significance level (<0.05) (adjusted RR = 1.069).

Finally, the health baseline incidence (*Y*_0_) is an estimate of the typical number of fatalities in a particular year (U.S. EPA, 2018). It was calculated from the ratio of the number of cases of mortality from respiratory diseases to the total population, as listed in Table 3. The *Y*_0_ was estimated using the following equation:

(3) $$\begin{array}{c} Y_{0}=\frac{Number\;of\;cases}{Total\;population}\text{.} \end{array}$$

## 3. Results and Discussion

### 3.1. Concentration of PM_10_ in Northern Thailand

Figure 2 illustrates the monthly average of PM_10_ concentrations from eight locations in the study areas. Most of the time, the concentration of daily PM_10_ in northern Thailand did not exceed the daily standard set by the Pollution Control Department (PCD), which is 120 *μ*g/m^3^. However, the results suggest that there was a 300 *μ*g/m^3^ spike reported in the study areas in March. This is because of the huge amount of biomass that is burned in northern Thailand [44] Furthermore, the influence of transboundary particulate emissions from surrounding countries, such as Myanmar and Laos, might boost the peaks of PM_10_ [11]. The decrease in PM_10_ concentrations for the eight stations begins in April and ends in November. It increased somewhat in December. The low PM_10_ concentrations in July and August were caused by the high rainfall rates across northern Thailand, where the southwest monsoon was active. Precipitation and deposition can wipe away particulate matter that is suspended in the atmosphere. The annual average PM_10_ concentration (Figure 3) ranged from 43 to 61 *μ*g/m^3^, with the highest and lowest concentrations of 61 and 43 *μ*g/m^3^, respectively.

### 3.2. Descriptive Analysis

Table 4 shows a descriptive analysis of the studied population's demographic characteristics, hospital admission outcomes, mortality rate from respiratory disease, and the average PM_10_ concentration in 2012 in northern Thailand. In 2012, a total of 83353 respiratory disease patients were admitted to inpatient departments (IPD) in northern Thailand. The WHO guidelines state that the annual PM_10_ concentration should not exceed 15 *μ*g/m^3^ (https://apps.who.int/iris/bitstream/handle/10665/345329/9789240034228-eng.pdf) and 50 *μ*g/m^3^ is Thailand's standard (https://www.pcd.go.th/wp-content/uploads/2021/10/pcdnew-2021-10-28_04-12-33_133858.pdf). In 2012, the average PM_10_ concentrations significantly exceeded the WHO standards for all provinces, falling in the range of 42–54 *μ*g/m^3^. Simultaneously, Thailand's standards were exceeded in Chiang Mai, Phayao, and Phrae, with concentrations of 53, 52, and 54 *μ*g/m^3^, respectively. Peaks of admission to IPD for respiratory disease exacerbation were registered in Chiang Rai, Nan, and Mae Hong Son for 2012 (Table 4). When considering the total population, the Nan and Mae Hong Son provinces had the highest IPD admission rates, with values of 2.57% and 4.35%, respectively. The mortality rate from respiratory disease was in the range of 0.26–0.40.

The exceeding of standard PM_10_ concentrations was likely associated with an increase in the risk of respiratory disease-related hospital admissions which is similar to that reported by Pini et al. [45] who reported that an increase in short-term exposure to particulate matter (PM_2.5_ and PM_10_) was strongly associated with a higher risk of emergency department (ED) admission and hospitalization. The highest mortality rate was found in Phayao province, with a value of 0.40, while Chiang Rai and Lampang also had high mortality rates, with values of 0.37 and 0.34, respectively. When we addressed a specific respiratory disease, there were high IPD rates from chronic lower respiratory diseases in those provinces, with values of 38.52%, 40.99%, and 43.87% in Phayao, Chiang Rai, and Lampang provinces, respectively. Chronic lower respiratory disease was associated with an increase in mortality related to PM_10_, along with chronic obstructive pulmonary disease and pneumonia [46].

### 3.3. Health Impact Assessment

Table 5 presents the avoided mortalities from respiratory diseases due to PM_10_ exposure in northern Thailand. In eight provinces of northern Thailand, the avoided impacts in terms of respiratory mortality of a daily mean concentration of PM_10_ were in the range of 2–18 (95% CI: 1–30) cases per year (rollback to 120 *μ*g/m^3^) and 4–47 (95% CI: 1–76) cases per year (rollback to 45 *μ*g/m^3^). When the daily PM_10_ concentration was reduced to 120 *μ*g/m^3^, the attributable risk percentage for respiratory disease mortality decreased by 1%–5%. When PM_10_ concentrations were reduced to 45 *μ*g/m^3^, the attributable risk percentage for respiratory disease mortality in northern Thailand changes from 1% to 12%.

The Health Impact Assessment for northern Thailand indicated that reducing the annual mean levels of PM_10_ would result in significant health benefits. Notably, complying with WHO-AQG for PM_10_ (45 *μ*g/m^3^) would result in substantial reductions in respiratory disease mortality. The number of preventable fatalities doubles with a reduction scenario level of 45 *μ*g/m^3^ compared to a reduction scenario level of 120 *μ*g/m^3^. This result is comparable to that of other studies, such as [47], who evaluated the annual health implications of particulate matter (PM) by reducing the annual mean PM_10_ concentration to 20 *μ*g/m^3^ in 27 cities in Southeast and East Asia in 2009. Although the second scenario of compliance reduction differs from Yorifuji et al. [47], the results of an 8% reduction in mortality in 27 Southeast and East Asian cities are comparable.

PM_10_ has an effect on respiratory illness mortality; however, other pollutants, such as NO_2_, PM_2.5_, O_3_, and CO, are also associated with respiratory mortality. Pothirat et al. [38] revealed that PM_2.5_ was related to acute exacerbations of chronic obstructive pulmonary disease (AECOPD), while CO, O_3_, and SO_2_ were related to visits to the emergency room (ER) for community-acquired pneumonia (CAP). Meanwhile, O_3_, NO_2_, and SO_2_ were correlated with heart failure (HF), myocardial infarction (MI), and cerebrovascular accident (CVA), respectively. According to the WHO [48], levels of PM exposure in Asian cities vary substantially. Nonetheless, the HIA analysis indicated that air pollution had a significant effect on public health in areas with comparatively high levels of air pollution and sizable populations. This conclusion implies that the public health implications of air quality in metropolitan areas with low to moderate exposure levels should not be disregarded. From a public health perspective, our estimates show that reducing PM_10_ concentrations in northern Thailand by 45 *μ*g/m^3^ is insufficient and that they must be decreased to the WHO-AQG. Here, only PM_10_ is considered; however, HIA-AQ can be used to assess the health effects of other pollutants. Future works should include other air pollutant data, such as ozone and PAHs, and place greater emphasis on fine PM and its components.

## 4. Conclusion

The purpose of this study was to analyze the annual health effects of particulate matter (PM) less than 10 *μ*m in diameter (PM_10_) in northern Thailand in the year 2012. The BenMAP-CE program was used as a tool for evaluating the health impact of PM_10_ in northern Thailand. PM_10_ concentration data collected from the Pollution Control Department (PCD) were used as the input data for BenMAP-CE. The results show that the annual average PM_10_ concentration was in the range of 43–61 *μ*g/m^3^, with a peak-observed PM_10_ concentration of 300 *μ*g/m^3^ in March. We further evaluated the effects of PM_10_ exposure in northern Thailand and found that, when the PM_10_ concentration is reduced to 120 *μ*g/m^3^, the effects on respiratory mortality tend to decrease by up to 5%. When the PM_10_ concentration was decreased to 45 *μ*g/m^3^, the adverse effects on respiratory mortality were reduced by up to 12%. According to the findings of this study, lowering the annual mean levels of PM_10_ would result in significant health benefits. Compliance with WHO-AQG for PM_10_ (45 *μ*g/m^3^) would result in significant reductions in respiratory disease mortality. Current air pollution levels in northern Thailand have a nonnegligible public health impact.

## Figures and Tables

**Figure 1:** Study area.

**Figure 2:** Monthly average PM_10_ concentrations across eight locations in northern Thailand in the year 2012.

**Figure 3:** Baseline daily PM_10_ concentrations in eight provinces in northern Thailand in the year 2012.

**Table 1:** PM_10_ observation data at eight locations in northern Thailand between 2010 and 2020.

Year	Percentage of missing data (%)	No. of days exceeding guidelines	Mean PM_10_ concentration (±SD)	Mortality rate
2010	14.40	170	47.5 (±8.8)	0.24
2011	15.10	6	35.4 (±4.2)	0.24
2012	8.60	175	47.6 (±4.4)	0.32
2013	20.10	156	47.3 (±4.3)	0.28
2014	5.80	171	46.6 (±5.7)	0.29
2015	7.40	136	43.1 (±4.9)	—^*∗*^
2016	3.80	145	44.1 (±3.7)	0.32
2017	4.20	30	35.9 (±4.3)	0.30
2018	8.30	33	36.1 (±3.4)	0.28
2019	6.30	114	44.7 (±7.6)	0.30
2020	0.80	125	44.9 (±2.8)	0.23

*Note*. ^*∗*^There was no mortality rate in 2015.

**Table 2:** Associations between PM_10_ and respiratory disease from COPD (adapted from [37]).

Outcomes COPD	PM_10_ adjusted RR (95% CI)
Lag 0	0.988 (0.943–1.035)
Lag 1	0.975 (0.933–1.019)
Lag 2	1.011 (0.963–1.063)
Lag 3	0.984 (0.930–1.035)
Lag 4	0.979 (0.928–1.042)
Lag 5	1.015 (0.972–1.033)
Lag 6	1.069 (1.017–1.123)^*∗*^
Lag 7	1.029 (0.990–1.069)

*Note*. ^*∗*^Statistical significance level < 0.05.

**Table 3:** The total population and mortality from respiratory diseases in northern Thailand in the year 2012 (https://service.nso.go.th/nso/web/statseries/statseries01.html).

Province	Population (million)			Mortality from respiratory causes (people)	
	All ages	Male	Female	Male	Female
Chiang Mai	1.65	0.80	0.84	289	187
Chiang Rai	1.2	0.59	0.60	212	166
Phayao	0.48	0.23	0.25	114	55
Nan	0.47	0.24	0.23	91	41
Mae Hong Son	0.24	0.12	0.12	23	13
Phrae	0.45	0.22	0.24	65	26
Lamphun	0.40	0.19	0.20	55	15
Lampang	0.75	0.37	0.38	133	81

**Table 4:** Descriptive analysis of the study population, mortality rate, hospital admission outcomes, and PM_2.5_ concentration in 2012 in northern Thailand.

Province	Population (million)			Hospitalization from respiratory disease (% = hospitalization/total population)	Hospitalization from respiratory disease			Mortality rate from respiratory diseases	PM_10_ concentration (*μ*g/m^3^)
	Male	Female	Total		Acute upper respiratory infections and other diseases of the upper respiratory tract	Chronic lower respiratory diseases	Other diseases of the respiratory system		
Chiang Mai	0.80 (48.48%)	0.84 (50.91%)	1.64	6138 (0.37%)	1169 (19.05%)	452 (7.36%)	4517 (73.59%)	0.32	53
Chiang Rai	0.59 (49.17%)	0.61 (50.83%)	1.20	23164 (1.93%)	4277 (18.46%)	9494 (40.99%)	9393 (40.55%)	0.37	42
Phayao	0.23 (47.92%)	0.25 (52.08%)	0.48	8655 (1.80%)	2507 (28.97%)	3334 (38.52%)	2814 (32.51%)	0.4	52
Nan	0.24 (51.06%)	0.23 (48.94%)	0.47	12070 (2.57%)	1891 (15.67%)	5702 (47.24%)	4477 (37.09%)	0.33	44
Mae Hong Son	0.12 (50.00%)	0.12 (50.00%)	0.24	10448 (4.35%)	4385 (41.97%)	3317 (31.75%)	2746 (26.28%)	0.3	44
Phrae	0.22 (48.89%)	0.24 (51.11%)	0.46	6933 (1.54%)	2022 (29.16%)	3611 (52.08%)	1300 (18.75%)	0.27	54
Lamphun	0.19 (47.50%)	0.20 (52.50%)	0.39	6067 (1.52%)	1809 (29.82%)	2076 (34.22%)	2182 (35.97%)	0.26	46
Lampang	0.37 (49.33%)	0.38 (50.67%)	0.75	9878 (1.32%)	1621 (16.41%)	4333 (43.87%)	3924 (39.72%)	0.34	47

**Table 5:** Mean estimated avoided mortality (95% confidential interval) from respiratory diseases in northern Thailand.

Province	Mortality from respiratory diseases	Roll back to 120 *μ*g/m^3^	Roll back to 45 *μ*g/m^3^	Attributable fraction (rollback to 120 *μ*g/m^3^) (%)	Attributable fraction (rollback 45 *μ*g/m^3^) (%)
Chiang Mai	476	9 (2–16)	40 (11–67)	2	11
Chiang Rai	378	18 (5–30)	47 (13–76)	5	12
Phayao	169	6 (2–11)	20 (5–33)	2	5
Nan	132	2 (1–4)	11 (3–19)	1	3
Mae Hong Son	36	2 (1–4)	4 (1–7)	1	1
Phrae	91	2 (1–4)	12 (3–19)	1	3
Lamphun	70	2 (1–3)	8 (2–13)	1	2
Lampang	214	7 (2–11)	22 (6–37)	2	6

## Data Availability

The data generated or analyzed during this study are included within the article. The observation data used in this study were provided with permission by the Pollution Control Department (PCD) for pollution data and the Department of Disease Control (DDC) of Thailand for mortality data and hence cannot be made freely available. Access to these data can be obtained by contacting the PCD at https://www.pcd.go.th/ and DCC at https://ddc.moph.go.th.
